# Multiorientation Simultaneous Computation of Back-Projection CT Image Reconstruction Algorithm in Staging Diagnosis of Bladder Cancer

**DOI:** 10.1155/2022/6731491

**Published:** 2022-06-28

**Authors:** Kaiyan Hu, Jianping Zhu, Pei Li, Lili Ying

**Affiliations:** Medical Imaging Center, Ningbo Yinzhou Second Hospital, Ningbo, 315100 Zhejiang, China

## Abstract

The objective of this research was to investigate the multidirectional synchronous calculation of the back-projection computed tomography (CT) image reconstruction algorithm (MSBP) in the staging diagnosis of bladder cancer. Sixty patients with bladder cancer admitted to the hospital were selected for enhanced CT scanning, all of which were randomly divided into control group (*n* = 30) and study group (*n* = 30). The filtered back-projection (FBP) algorithm was employed to reconstruct the scanned image, and the MSBP was additionally applied to the images of the study group. Fringe artifact (SA), overall mass (OQ), effective radiation dose (ED), CT dose-exponential volume (CTDI), and dose-length product (DLP) of the two groups of images were compared and analyzed. The results showed that the total time of the traditional algorithm was 5.473 s, and the total time of MSBP combined with FBP algorithm was 2.832 s, which was significantly higher than that of the traditional algorithm (*P* < 0.05). CT scan bladder cancer staging results of all patients were compared with surgical pathological staging results, and the results were evaluated according to the coincidence rate. SA in the study group was lower than that in the control group (*P* < 0.05), and OQ was not statistically significant. The ED of the study group was significantly lower than that of the control group by 33%. The coincidence rate of postoperative pathological staging results and CT staging results was 96%, and T1, T2a, and T4 coincidence rate was 100%, The coincidence rates of T2b, T3a, and T3b were 90%, 83.3%, and 66.67%, respectively. In summary, using MSBP method combined with FBP algorithm can improve OQ while reducing ED of patients. The introduction of MSBP into CT reconstruction image simplified the pixel location operation of projection calculation, showing an important application value in preoperative staging diagnosis of bladder cancer.

## 1. Introduction

With people's attention to health and the development of clinical diagnosis technology, the number of new cases of bladder cancer is increasing year by year [1–3]. Bladder cancer often involves transitional epithelial carcinoma, which is prone to occur at the lateral wall of the bladder and the trigone near the ureter opening and is prone to recurrence. Cystoscopy and biopsy are the gold standard for bladder cancer [4, 5]. Understanding the pathological stages and lesion sites of bladder cancer as soon as possible has a good reference value for the early development of targeted diagnosis and treatment plan and prognosis. CT scanning is currently a noninvasive imaging method for patients with bladder cancer [6, 7]. It can not only quickly display bladder tissue but also obtain the maximum scanning range in one scan, which can provide reliable information for clinical judgment of bladder cancer stage type. Although the advantages of CT scans can help bladder cancer patients obtain more accurate lesions, patients must bear the risk of radiation during the scan. The effective radiation dose (ED) is related to the quality of CT scan image. To some extent, when ED is increased, the image quality is better [8]. Therefore, after accurate CT scan image quality of patients is improved, how to minimize radiation risk is the focus of current medical researchers. In recent years, with the updating of computer technology, many researchers found that image reconstruction algorithms can be used to reduce the radiation risk of CT scanning [9].

CT image reconstruction technology solves the pixels in the image matrix according to the collected data, and filtering back-projection algorithm can collect features of images in the process of image reconstruction and is widely used in CT reconstruction technology [10]. Filtering back-projection algorithm is also called convolution back-projection algorithm. Before back-projection, the projection under each acquisition projection angle is convolved, so as to improve the shape artifact caused by point diffusion function and reconstruct the image with good quality. Filtering back-projection is easy to be implemented by software and hardware and can produce accurate and clear images with high data quality. Some scholars reconstructed multiorientation simultaneous computation of back-projection (MSBP) between image pixels and projection rays in different projection directions [11]. In the processing of CT images, MSBP algorithm can be used for rapid calculation in the space domain of direct back-projection, further reducing the amount of calculation in pixel positioning operation [12–14]. At present, there are very few data to apply HIR algorithm to CT scan images of bladder cancer patients. Therefore, this study intended to perform the multislice spiral CT (MSCT) scans of different doses for patients with bladder cancer and then processed the original images obtained through the HIR algorithm to compare the processed image quality, aiming to analyze the application of MSCT scans in the staging diagnosis of bladder cancer.

## 2. Methods

### 2.1. Research Objects

Sixty patients with bladder cancer who were admitted to the hospital from April 2018 to February 2021 were selected for MSCT scan. There were 43 male patients and 17 female patients. All patients were 42-79 years old, with an average of 60.5 years old. 30 patients were randomly selected to scan at 120 kV and 250 mAs and set as the control group, and 30 patients were scanned at 100 kV and 225 mAs to set the study group. All patients and their authorized persons in this study had signed the informed consent forms, and this study had been approved by ethics committee of hospital.

Inclusion criteria were as follows: patients whose diagnosis result was bladder cancer according to *the 2021 version of Chinese Guidelines for the Diagnosis and Treatment of Bladder Cancer* [15]; patients who could accept the CT scans with no allergic contraindication to contrast agents; patients whose routine laboratory examinations before scanning confirmed that the bladder tumor was the primary lesion without metastasis; and patients who were the initial diagnosis and treatment.

Exclusion criteria were as follows: patients with a history of radiotherapy and chemotherapy; patients with other acute infectious diseases; patients whose bladder cancer was more serious, and the tumor had metastasized to other tissues; and patients with mental and consciousness disorders and poor compliance.

### 2.2. CT Examination

64-slice spiral CT scanner was used. All patients started fasting hours before the operation, and within 1 hour before the CT scan, the patients' bladder was filled by drinking 500 mL of water. The scanning range was from the top of the patient's bladder to the lower edge of the symphysis pubis, with a thickness of 5 mm and a distance of 5 mm. Scanning parameters were set as follows: in the control group, the tube voltage was 120 kV and the tube current was 250 mAs; in the research group, tube voltage was 100 kV, and the tube current was 225 mAs. The rotation speed of the bulb was set to 2 revolutions per second; iohexol was selected as the contrast agent, injected with a high-pressure CT syringe at a flow rate of 3 mL/s, and the dose was 100 mL. In addition, an enhanced scan was performed on the lesion area in 60 s, and then, a delayed scan was performed after 3 to 5 minutes. In the CT examination, patients in the control group performed conventional CT imaging, and the FBP algorithm was induced in the study group to perform CT imaging of the patients.

### 2.3. Back-Projection Reconstruction Algorithm

The back-projection reconstruction algorithm is also called linear superposition method, summation method, and accumulation method. In the total projection reconstruction image algorithm, the density of a point in the fault plane can be regarded as the sum of the ray projections of all the changed points within this square meter in the simplest and most basic algorithm.

In the process of tomography, the X-ray tube moves from left to right, the film moves in the opposite direction, and the X-ray intensity *W* acting on the film is related to the corresponding ray projection *P*.

(1) $$\begin{array}{c} P=\int_{L}\mathrm{\mu dl}-\text{In}\frac{w_{0}}{w}. \end{array}$$

X ray intensity *I* causes the change of film transmittance *Q*Δ*Q*, and the change degree of film blackening is as follows.

(2) $$\begin{array}{c} \frac{\Delta Q}{Q}=\varphi In\frac{w_{0}}{w}, \end{array}$$

where *φ* is the contrast coefficient of film, and equations (1) and (2) are combined to the following equation.

(3) $$\begin{array}{c} \frac{\Delta Q}{Q}=\varphi P. \end{array}$$

There is a point *D* on the plane, and the density of the body tissue is set as *f*(*x*, *y*, *z*), denoted by the *n*-th projection of point *D*.

(4) $$\begin{array}{c} \text{P}\mu =\int_{L_{N}}\text{f}\left(x,y,z\right)\text{dl}. \end{array}$$

The changes in transmittance caused by the projection are added together to form an enhanced image of point *D*.

(5) $$\begin{array}{c} \underset{\text{i}}{\sum }\left(\frac{\Delta Q}{Q}\right)\mu =\varphi \underset{\text{i}}{\sum }p\mu , \end{array}$$

where ∑_i_*pμ* represents the sum of all ray projections through point *D* and *φ* is a constant. The above equation represents the idea of image reconstruction by back-projection.

Figure 1 is the fault parallel to the plane, with 16 pixels, each pixel value is *X*1, *X*2 ⋯ *X*16, and the reconstructed pixel value after assignment is shown in the figure.  Figure 2(a) is the original pixel value, and Figure 2(b) is the pixel value after back-projection reconstruction shown in Figure 2(c) divided by the number of pixel projections. After back-projection reconstruction, points with zero-pixel value in the original image are more prominent, but no longer zero after back-projection reconstruction.

### 2.4. Filtering Back-Projection Reconstruction Algorithm

The back-projection reconstruction algorithm introduces star artifact; that is, the point with zero density in the original image will not be zero after reconstruction, which is called image distortion. The filtering back-projection reconstruction algorithm can modify the projected data, and the modified projection data can be back-projected to obtain the image without artifact. The specific artifact removal flow chart is shown in Figure 3.

The position of point (*x*_*r*_, *y*_*r*_) in the image coordinate system is expressed by the following equation.

(6) $$\begin{array}{c} \text{f}\left({\text{x}}_{r},y_{r}\right)=\frac{1}{N_{\psi }}\overset{N_{\psi }}{\underset{i=1}{\sum }}p_{\psi }\left(x_{r}\right). \end{array}$$

where *N*_*ψ*_ is the projection number.

To find all rays passing through the modified point at any point (*r*, *g*), the mean projection of the rays at the modified point can be obtained. The 2D Fourier transform of *t*(*x*, *y*) is

(7) $$\begin{array}{c} T\left(\omega 1,\omega 2\right)=\hat{T}\left(\rho ,\theta \right). \end{array}$$

Agent construction image is as follows.

(8) $$\begin{array}{c} \hat{T}\left(\rho ,\theta \right)=T\left(\text{x},y\right)=\int_{0}^{x}\int_{-\infty }^{\infty }p\left(\rho ,\psi \right)e^{2\pi \text{pr}\cos\left(\theta -\psi \right)}\left|\rho \right|dpd\psi . \end{array}$$

Filtering back-projection centrally reflects each step of filtering convolution back-projection algorithm and finally obtains the reconstructed image.

The purpose of using a filter is that the filter function is hoped to have a high accuracy. Giving that the data in the process of projection is naturally discrete, the amplitude of high-frequency component is small and there is noise; it needs to be processed by filtering function. The selected window function *W*(*P*) can alleviate the oscillation response and complement the mixing better. The system function equation is as follows.

(9) $$\begin{array}{c} H_{S-L}\left(\rho \right)=\left|\rho \right|\sin c\left(\rho /2B\right)\text{rect}\left(\rho /2B\right)=\left|\frac{2B}{\pi }\sin\frac{2B}{\pi }\right|\text{rect}\left(\rho /2B\right). \end{array}$$

The image reconstructed by *S*‐*L* filter function has reduced oscillation response and better reconstruction quality of noisy data than *R*‐*L* filter function, but the reconstruction quality of low frequency is not as good as *R*‐*L* filter function.

If there is a rotation angle, projection *P*(*x*) is used, the filtering function is *H*(*xr*), and the filtered projection is expressed as follows.

(10) $$\begin{array}{c} \bar{P}\left(\text{x}r,\varphi_{m}\right)=\int_{-\infty }^{\infty }p\left(x_{r}-x\prime_{r}\right)h\left(x\prime_{r}\right)dx\prime_{r}. \end{array}$$

### 2.5. General Theorem of MSBP

In the *xoy* plane, there is a parallel line with equal intervals, numbered in a certain way, which rotates about the point *O*(*X*, *Y*) of rotation at an angle of rotation *φ*. The geometric position of the straight line set when the rotation angle is 0 in the XOY system is shown as the parallel line of *y*-axis. *dr* is the cluster of the nearest straight line from *O* to the right. *L* is the interval between two adjacent lines. For any rotation angle *dr* = 0 or *dr* = *L*/2, we have the following equation.

(11) $$\begin{array}{c} \text{d}\varphi \left(x,y;i_{p}\right)=d\varphi \left(-x+2x_{0},-y+2_{y}0;i_{n}\right). \end{array}$$

MSBP can simplify the pixel location operation in the back-projection. The network of the target image must be properly arranged so that the matching point of a pixel is also the pixel of the image to select a certain grid of the target image, and the origin coordinate position of the target image should be appropriately selected. A simple case is that the origin of the rotating point threshold target image is overlapped and a ray passes through the rotating center.

### 2.6. Image Evaluation Indicators

Two experienced professional imaging doctors were invited to qualitatively evaluate the obtained images *y* taking overall quality (OQ) and streak aircraft (SA) as indicators. The full score was specified as 10 points. The higher the score, the less noise and the better the image quality. The effective radiation dose (ED), CT dose index volume (CTDI), and dose-length production (DLP) were selected to evaluate the ED received by the patient.

### 2.7. Pathological Evaluation Indicators

The pathological evaluation was evaluated by two radiology clinicians. The staged diagnosis was based on the spiral CT scan results before the surgery, and the pathological results were used as the standard for the staged diagnosis after the surgery. The evaluation criteria for staging of bladder cancer were based on the 2020 version of *TNM Staging Standards*: T0 means no primary tumor; T1 means that the tumor mainly infiltrates the subcutaneous tissue; T2a indicates that the tumor infiltrates the superficial muscle layer, T2b indicates that the tumor infiltrates the deep muscle layer; T3a indicates that the tumor infiltrates the tissue around the bladder under the microscope; T3b indicates that the tumor infiltrates the tissue around the bladder by naked eyes; and T4 tumor has infiltrated the organs around the bladder, such as the pelvis and prostate.

### 2.8. Statistical Analysis

All data in this study were analyzed by SPSS20.0 statistical software; and the difference between groups was analyzed by the chi-square test method. The analysis method was selected according to different situations, and the measurement data that conformed to the normal distribution were expressed as mean ± standard deviation ($\overset{¯}{x}\pm s$). The *t* test was used for the comparative study of the index samples. Enumeration data were tested by *χ*^2^. General demographic data were described using frequency, percentage, mean, standard deviation, etc. When *P* < 0.05, it meant that the difference was statistically significant.

## 3. Results

### 3.1. Basic Information of the Two Groups of Patients

The general clinical data of patients in the control group and the study group are shown in Table 1. The two groups of patients showed no obvious differences in gender, age, and body mass index (BMI), and they were comparable.

### 3.2. Evaluation Results of Scanned Image

The timer of MATLAB was used to conduct the calculation time statistics of pixel positioning, interpolation operation, and back-projection of the algorithm. The results are shown in Figure 4. The total time of the traditional algorithm was 5.473 s, and that of the reconstruction algorithm was 2.832 s, which was significantly higher than that of the traditional algorithm (*P* < 0.05).  Figure 5(a) is the original image (52-year-old male patient presented with a large irregular filling defect in the anterior wall of the bladder roof due to repeated terminal gross hematuria for more than 1 year). Figures 5(b)–5(d) show the reconstructed image after S-L filtering function, R-L filtering function, and MSBP method. The reconstructed image was obviously clearer than the original image.

### 3.3. Image Quality Evaluation Results

The OQ and SA of the image were independently scored and evaluated by two professional imaging doctors. The results are shown in Figure 6. In the scoring results of the two imaging doctors, the SA of the control group was different from that of the research group (*P* < 0.05). The SA of the study group was lower than that of the control group. In addition, the OQ scores given by two doctors for the research group were higher than those for the control group, but they were not statistically significant.

### 3.4. Assessment Results of ED

The evaluation results of the two groups of ED are shown in Figure 7. Compared with the control group, the three ED parameters of the research group were observably reduced (*P* < 0.05). The ED of the research group was 2.58 ± 1.67, and the ED of the control group was 7.89 ± 1.43. The ED of the research group was much lower than that of the control group by 33%.

### 3.5. Comparison on CT Staging Results of Bladder Cancer with Postoperative Pathological Staging

The CT staging results and postoperative pathological results of 60 bladder cancer patients are shown in Table 2 and Figure 8. The postoperative pathological staging results were as follows. There were 3 cases in T1 stage, 25 cases in T2a stage, 22 cases in T2b stage, 5 cases in T3a stage, 2 cases in T3b stage, and 3 cases in T4 stage. The results of CT staging proved there were 3 cases in T1 stage, 25 cases in T2a stage, 20 cases in T2b stage, 6 cases in T3a stage, 3 cases in T3b stage, and 3 cases in T4 stage. The coincidence rate of postoperative pathological staging results and CT staging results was 96% (58/60). The coincidence rates of T1, T2a, and T4 were 100%, and those of T2b, T3a, and T3b were 90%, 83.3%, and 66.67%, respectively.

## 4. Discussion

CT can judge the tumor size, damage of surrounding organs, lymph node status, and invasion depth during preoperative examination of bladder cancer. Introducing intelligent algorithm into CT imaging can greatly improve the sharpness of image [16]. Jing et al. [17] can clearly supervise the training process of fuzzy images by using 3D reconstructed CT images, and the intelligent algorithm used showed good results. Huang et al. [18] used intelligent algorithm to ensure the quality of CT image registration and obtain the accuracy of dual-energy images. In this study, the intelligent algorithm was applied in CT imaging to explore the bladder cancer staging. After the algorithm was introduced, a clearer image can be obtained. When MSBP was added into CT images of patients in the study group, the total time of MSBP method combined with filtering back-projection algorithm was 2.832 s, significantly higher than that of the traditional algorithm (*P* < 0.05). Preoperative classification of bladder cancer also had certain influence on the analysis of pathological changes, and it was difficult for surgeons with different experience to distinguish the classification. Patients under local anesthesia who do not cooperate during surgery and the number of samples collected will inevitably be like the preoperative biopsy grading.

The introduction of intelligent algorithms in CT imaging has effectively improved the image quality. Liu et al. [19] adopted the adaptive statistical iterative reconstruction algorithm, which showed the characteristics of high noise degree, few artifacts, and good overall quality in CT images, which was of great significance for clinical diagnosis. This study is consistent with its findings. Valencia Pérez et al. [20] reconstructed CT images based on the maximized iterative algorithm, which showed good performance. The image quality and reconstruction time were not affected by the noise in the projection. In this study, after the reconstruction of CT images by MSBP, the bladder lesions became clearer, and the resolution and quality of the images were also improved. The total construction time of the algorithm in this research was 2.832 s, which was significantly higher than the traditional algorithm. The image obtained after reconstruction was clearer. It was found that the filtering back-projection reconstruction algorithm can reduce the estimated radiation dose while maintaining the image quality. The ED of the study group was significantly lower than that of the control group.

At present, CT scan is a better imaging examination mean for the diagnosis of bladder cancer. Its main value lies in staging, which can observe the scope and extent of tumor accumulation in the bladder and can also show the invasion of adjacent organs and the presence or absence of lymph node and distant metastasis [21, 22]. The results in this work showed that CT was better than B-ultrasound in diagnosing bladder cancer, the accuracy of CT staging was 96%, and the images displayed by CT scan images were clearer. Helenius et al. performed CT examinations on the histological types of bladder cancer patients, indicating that CT scan can better help patients with bladder cancer for accurate staging diagnosis [23]. Yang et al. performed CT scan staging and postoperative pathological staging on bladder cancer patients and compared the staging diagnosis results of bladder cancer on CT scans and the staging results of bladder cancer in surgical pathological examinations [24]. The results of this study also found that, compared with the pathological diagnosis results, CT scan showed a 100% coincidence for T1 staging diagnosis, T2 staging diagnosis had a 95% coincidence, and the coincidence rates of diagnosis for stages T3 and T4 were 75% and 100%, respectively. The coincidence rate of overall postoperative pathological staging results and CT staging results was 96%.

## 5. Conclusion

In this research, MSBP was applied to the CT image back-projection reconstruction algorithm to analyze the CT images of bladder cancer patients. The CT image reconstructed by FBP was clearer, which can accurately diagnose the preoperative staging of bladder cancer, and the CT image clearly showed the location of the lesion. Intelligent CT images based on FBP algorithm had certain application value for the diagnosis and staging of bladder cancer and were worthy of clinical promotion. There were still some deficiencies in this research. For the training of intelligent algorithms, how to design filter functions to obtain stronger image smoothness can be considered in the future. All in all, the MSBP-based back-projection reconstruction algorithm in CT images can improve the image quality and be able to diagnose bladder cancer staging.

## Figures and Tables

**Figure 1:** Fault pixel values and rays.

**Figure 2:** The result of back-projection reconstruction.

**Figure 3:** Artifact removal flow chart.

**Figure 4:** Comparison of computation amount of pixel operation between different algorithms. ∗ meant statistically significant difference, *P* < 0.05.

**Figure 5:** CT image of a patient with bladder cancer.

**Figure 6:** The scoring results of two groups. (a) showed the OQ scoring results of the first doctor; (b) showed the scoring result of the first doctor on SA; (c) showed the scoring result of the second doctor on OQ; and (d) showed the scoring result of the second doctor on SA. ∗ meant the difference between research group and control group was statistically obvious (*P* < 0.05).

**Figure 7:** Evaluation results of ED in the two groups. ∗ meant *P* < 0.05.

**Figure 8:** CT scan images of bladder cancer staging effects. (a)~(d) showed the images in stages T1, T2, T3, and T4, respectively.

**Table 1:** Comparison on general information of the two groups of patients.

Group	Gender (male/female)	Age (years old)	BMI (kg/m^2^)
Control group	26/9	59 ± 3.1	23.34
Study group	17/8	60 ± 1.7	24.53
*P* value	0.492	0.964	0.712

**Table 2:** Comparison on CT staging results and postoperative pathological staging results.

Pathological staging results	CT staging results						Total
	T1	T2a	T2b	T3a	T3b	T4	
T1	0	0	3	0	0	0	3
T2a	0	14	6	5	0	0	25
T2b	3	9	8	0	2	0	22
T3a	0	0	2	1	0	2	5
T3b	0	2	0	0	0	0	2
T4	0	0	1	0	1	1	3
Total	3	25	20	6	3	3	60

## Data Availability

The data used to support the findings of this study are available from the corresponding author upon request.
